The article "Inventorization of traditional ethnobotanical uses of wild plants of Dawarian and Ratti Gali areas of District Neelum, Azad Jammu and Kashmir Pakistan" was retracted in 2023. Reasons: a conflict of interest; concerns about the peer review; concerns about the authorship.

# Inventorization of traditional ethnobotanical uses of wild plants of Dawarian and Ratti Gali areas of District Neelum, Azad Jammu and Kashmir Pakistan

**DOI:** 10.1371/journal.pone.0255010

**Published:** 2021-07-29

**Authors:** Muhammad Ajaib, Muhammad Ishtiaq, Khizar Hayat Bhatti, Iqbal Hussain, Mehwish Maqbool, Tanveer Hussain, Waheeda Mushtaq, Abdul Ghani, Muhammad Azeem, Sardar Muhammad Rafique Khan, Sumaira Thind, Rohina Bashir

**Affiliations:** 1 Department of Botany, Mirpur University of Science and Technology (MUST), Mirpur, Azad Jammu and Kashmir, Pakistan; 2 Department of Botany, University of Gujrat, Gujrat, Pakistan; 3 Department of Botany, Government College University, Faisalabad, Pakistan; 4 Department of Botany, University of Sargodha, Sargodha, Pakistan; 5 Department of Climate Change Centre, Environmental Protection Agency, AJK, Muzaffarabad, Pakistan; University of Poonch Rawalakot, PAKISTAN

## Abstract

**Background:**

An ethnobotanical expedition was conducted to document the traditional ethnobotanical (TEB) uses of wild flora of Dawarian and Ratti Gali villages of District Neelam, Azad Jammu and Kashmir (AJK) Pakistan. District Neelam has rich plant diversity and is hub of many endemic plant species while the study areas are not yet explored. The research area: Dawarian and Rati Gali (DRG) area is mountaineous terrain and villages are located on far and farther distances. DRG area has rich biocultural and plant diversity comprising of different ethnic groups of Kashmir state. The current research was aimed to explore and document traditional medicines (TEMs) and other domestic and commercial uses of wild plants. This study will assist to evaluate conservation and commercial worth of wild flora which can be potential candidate for drug discovery through ethnopharmacological analysis.

**Methods:**

The current quantitative ethnobotanical research was carried out in 2018 by interviewing 150 indigenous informants (90 male and 60 female) of DRG area using questionnaire applying structured and semi structured interview methodology. Data analysis was analyzed by using quantitative ethnobotanical statistical tools such as fidelity level (FL), informant consensus factor (ICF), Spearman’s rank correlation (SRC) and data matrix ranking (DMR).

**Results:**

The indigenous people of DRG area use wild plants in their daily life to cope life necessities i.e. food, vegetables, fodder, fuel, shelter, timber and herbal medicines. TEMs are primarily used to cure different infirmities like diabetics, asthma, dysentery, constipation, cold, fever, joint pain, wound healing, cancer, cardiovascular disorders, epilepsy, kidney infections and many types of skin diseases. Current study revealed the data of 103 wild plants species belonging to 46 plant families from selected areas of District Neelum, AJK. Results depicted that Asteraceae ranked 1^st^ (12 plants spp). Among plant parts used leaf ranked 1^st^ (18%), followed by seed (17%) and root (13%). While prevalent form recipe mode was decoction (20%), followed by powder (17%) and extract (14%) and fodder was highest (37%) EB use-form fodder, followed by food (32%) and fuel (17%). Quantitative ethnobotanical analysis (QEA) was carried to find the reliability and novelty of the study. Five plant species including *Berberis lyceum* (FL = 97.78%), *Isodon rugosus* (FL = 95.71%), *Saussurea lappa* (FL = 94.74%), *Aconitum heterophyllum* (FL = 92.71%) and *Taxus baccata* (91.58%) had shown high fidelity level which confirmed that these plants have high medicinal worth in study area. The highest value (0.94) of ICF was for diseases group “tuberculosis and leucorrhea”, followed by stomachache and flatulence (0.93), diabetics and blood pressure (0.92) and asthma and chest infections (0.88). For other uses fuel with ICF (0.83) ranked first and second was hedging and thatching (ICF = 0.82) where people use plants or their parts for construction. Spearman’s rank correlation (SRC) test indicated that number of TEB uses increases if number of species is increased. Jaccard index (JI) analysis depicted that 56.31% plants are being used as TEMs which are first time explored from the study area. While 26.21% plants are being used in different TEB uses which are different from past cited literature. These novel findings of research indicate that wild flora of the study area has great potential for novel drug discovery and provision of materialist services for the indigenous communities.

**Conclusion:**

The present research revealed that TEMs uses of 58 plants are novel being first time reported from the study area (DRG) of District Neelam of AJK. The results showed that plants like *Acer cappadocicum*, *Ajuga bracteosa* and *Swertia paniculata* are used to cure diabetes, *Viscum album*, *Viola canescens*, *Taxus baccata* are used for cure of cancer, *Isodon rugosus*, *Polygala chinensis* are used in TEMs for treating cardiovascular disorders and *Anaphalis triplinervis* is used for epilepsy. *Berberis lyceum*, *Ajuga bracteosa*, *Aconitum heterophyllum*, *Bistorta amplexicaule*, *Saussurea lapa* and *Jurinea dolomiaea* are severely threatened and there is urgent need to do conservation measures for available of valuable MPs to the indigenous communities for life necessities and for future research. The current study will also be useful addition in ethnobotanical database, preservation of traditional culture and drug discovery and drug development through future ethnopharmacological research.

## Introduction

Plants are very indispensable for life sustenance because rural communities of different countries primarily use local plants in multiple forms. The ethnobotany roots back to era when first man started his life on this planet and he used wild natural resources for life necessities. Ethnobotany plays a significant role between biological diversity, social culture and traditional medicine system [1,2]. It is cited and proved that indigenous knowledge of ethnomedicinal uses of plants is usually transferred orally form one generation to other and there is risk of loss of biocultural and traditional ethnobotanical uses of wild indigenous plants (WIPs) [3]. Ethnobotanical study provides comprehensive information about cultural uses of plants as ethnomedicines, folklore food phytonyms, fodder, fuel, rituals usage and shelter [4]. The plants of medicinal worth have been used in novel drug discovery and development through ethnopharmacological analysis in previous. Furthermore, ethnobotanical study (EBS) is supportive and essential for knowledge based economy for research in other subjects like Biology, Agriculture and Pharmacology because EBS provides baseline data for further research [5]. WIPs are being used for different perspectives for existence of life activities according to their ethnicity and cultural paradigm around the globe [6]. In past research it is stated that 25% allopathic drugs are produced from plants or their byproducts and nearly 80% people of the world hitherto are dependent on TEMs obtained from fresh or dried plants or their products for cure of different diseases [7,8]. Many other necessary requirements of life such as shelter, forage, fodder, fuel, aesthetic use and fiber are gained from forests’ vegetation or other WIPs of in different regions of the world [9,10]. WIPs of any area generally provide fuel and timber wood which primarily fulfill basic need of life and on secondary level it also provides sources of livelihood to local communities through timber and furniture industry [11]. Many past studies are supporting the theme that plants are pivotal source of phytotherapeutic to cure of various human and veterinary diseases. The EBS reveals the conservation status of WIPs in an area and it is reported that *Berberis lyceum*, *Ajuga bracteosa*, *Aconitum heterophyllum*, *Bistorta amplexicaule*, *Saussurea lapa* and *Jurinea dolomiaea* are severely threatened and are on verge of extinction due to overgrazing, excessive harvesting for forage, fire, cutting by timber mafia, building of infrastructure and agriculture expansion for crop cultivation [12–17].

The study areas (Dawarian and Ratti Galli) are part District Neelam which is one of the administrative units of state of Azad Jammu and Kashmir (AJK). AJK has diverse habitats, variable climatic conditions and appropriate fertile soil endowed with plant biodiversity out of which some are endemic to this region [18–20]. The current study is focused on two rural areas (DRG) of Neelum valley which is present in North-East of Muzaffarabad with altitude of 900–6325 meters occurring between 73°-75° E longitude and 32°-35° N scope [21]. Neelam valley is the biggest vale of Azad Jammu and Kashmir (AJK) covering a territory of 3737 Km. Dawarian is its one of the towns with 110 km and Ratti Galli is at 75 Km distance north of Muzaffarabad city at altitude of 5299 ft from sea level (Fig 1). The atmosphere is chilling winter with temp. 0–4°C and summer with 18–25°C and precipitation is 1650 mm per annum. Soil of the area is loamy appropriate for holding dampness which makes it useful woodland with thick vegetation [22].

**Fig 1:** Map of Darian and Rati Gali, District Neelam of Azad Jammu and Kashmir, Pakistan (note: Study sites are encircled).

It is mentioned in many studies that flora of different areas of Neelam valley are under severe anthropogenic pressure and other natural catastrophe accelerate this more which do have a high impact on the ecosystems structure and services for the indigenous people [23]. Vegetation of DRG mainly consist of herbs and shrubs with some tree species. Ratti Gali is famous place because of lake known as “Ratti Gali lake” (RGL) which is an alpine glacial lake (Fig 1). RGL nearby areas have rich plant biodiversity due to altitude and rich moisture.

Many wild indigenous plants (WIPs) are being used source of food, vegetables and fruits. Many of WIPs are commonly used as source of fuel, fodder and forage for domestic animals [24]. The indigenous people of DRG areas use local WIPs as traditional ethnomedicines (TEMs) to cure various chronic and acute infirmities and similar is practised in the other areas of AJK [24]. The literature persual and field survey analysis depicted that older indigenous people of AJK territory has more ethnobotanical knowledge of WIPs as compared to young generation because former have strong belief on traditional and cultural customs and prefer plant-based drugs which they deem safe and economic in use [24].

It is first ethnobotanical study conducted on DRG areas of Neelam valley and only scarce literature is cited in some articles from other districts and some parts of NV of AJK. Many WIPs species of the study area were unexplored and here first time reported in this paper. The present research was focused ethnobotanical study in conjunction biocultural paradigms of indigenous ethnic groups along with geographical characteristics of different study sites encompassing on plant biodiversity. The key objectives of the study were to: (i) document biocultural data of traditions of indigenous communities, (ii) prepare floristic checklist of WIPs describing occurrence range, (iii) document ethnobotanical uses of WIPs, especially enlisting inventory of TEMs, (iv) on basis of ethnobotanical study, screening of potential medicinal plants for further phytochemical research and (v) determine their potential for drug discovery to combat multi-drug resistant (MDR) bacteria and other microbes. The research will also assist in conservation of precious WIPs of the area because they provides current population status of the species and key threats for plants of the study area.

## Materials and methods

The current ethnobotanical research study was conducted during the year 2019 from Dawarian to Rati Gali (DRG) sites of District Neelum of Azad Jammu and Kashmir, Pakistan. The area was selected to due to interesting reasons that (i) it is remote area located very far from main city, Muzaffarabad of AJK, (ii) diverse ethnic and biocultural diversity and rich plant biodiversity. Furthermore, the native people have traditional bioculture and customs primarily depend on wild plants for treatment of many diseases.

### Collection of ethnobotanical information

Traditional ethnobotanical (TEB) informations were gathered from local informants of the study area by using structured and semi-structured interview methodologies. The planned and random visits were made in the study and 150 informants (90 male and 60 female) with age range of 40-to-90 years were asked questions with assistance of local guide or translator. Prior to field visit of different mountaineous areas of DRG; the heads/leaders of villages were contacted and purpose of this study was informed to all participants. The privacy and secrecy of their personal and culture was promised to be kept intact (however, permission for using this valuable information for thesis writing and publishing it in article form was obtained verbally). The data collected from the local people included: local name, local uses, recipe, plant part used, occurrence, characters involved in the collection, marketing and other related information. The plants of two hilly villages of Dawarian and Rati Gali of District Neelum were categorized according to their economic value such as medicinal, food, fodder, vegetable, fruit, thatching, hedging, timber and fuel wood. The collected information was compiled and compared to relevant literature to evaluate the authenticity and explore novelty of knowledge [24]. For ethnopharmacological purpose, the interviewer were enquired that how a particular plant species was used, dosage form, part used and herbal recipe for treatment of prevalent diseases [25]. The protocol of Thompson [25], Ishtiaq *et al*., and Mehwish *et al*., [26,27] with some modifications were employed for TEB data collection and analysis.

The collected plants were properly dried, pressed and mounted on the herbarium sheets following standard protocol [26,27]. The each specimen was identified by expert taxonomist using Flora of Pakistan (from library) and a voucher number was assigned to each plant and submitted in herbarium (MUH) of Department of Botany, Mirpur University of Science and Technology (MUST), Mirpur AJK (Pakistan) for future reference. The identified taxa were cross checked and verified using online information of plant flora from “the plant list” web repository (http://www.theplantlist.org) and world flora www.worldfloraonline.org [19,26,27] and authticated plants were kept in herbarium according to proper procedure of herbarium.

### Data analysis

The collected data was tabulated and analyzed by using different quantitative ethnobotanical micro statistical tools i.e. fidelity level (FL), informant consensus factor (ICF), fidelity level (FL), family index (FI) and spearman’s rank correlation (SRC) were employed to find its novelty and authenticity of TEB and ethnomedicines [26,27].

#### Fidelity level (FL)

The fidelity level is the level of witnesses guaranteeing the utilization of certain plant for a similar object or purpose. FL describes how a plant is commonly or certainly used for curing of a specific disease or infirmity in the stud area. FL was determined by using follow equation as per protocol cited by Ishtiaq *et al*., and Mehwish *et al*., [26,27]:

$$\text{FL}\;\left(\%\right)\;=\;\text{Np}/\text{N}\times 100$$

where, Np indicates the number of informants that claim “a use of the plant species” used for “a particular purpose/disease” and N is mentioned “the number of informants” that use the plant as a medicine to treat any given disease.

#### Informants consensus factor (ICF)

ICF identifies the agreement of the informants on the reported herbal medicines for the cure of group of ailments. It was calculated by the following procedure of Ishtiaq *et al*., and Mehwish *et al*., [26,27] using following equation:

$$\text{ICF}\;=\;{\;\text{n}}_{\text{ur}}-{\;\text{n}}_{\text{t}}/{\text{n}}_{\text{ur}}-1$$

where, n_ur_ is “the number of use citation” in each category and n_t_ denotes “number of species used” to cure particular group of disease or diseases. The method is recommend for further exploration of drug using different ethnopharmacological approaches [28].

#### Family index (FI)

Family index is calculated to check which family has highest number plants being used as ethnomedicines to cure different diseases in the local communities of any study area [13,26,27].

#### Direct Matrix Ranking (DMR)

Direct matrix ranking is applied to find out populace thickness of plant species and their protection status in the investigation territory. DMR depicts highest biotic pressure on the plants which are predominantly used by local people in the investigated area for the treatment of various ailments [24,26,27].

#### Spearman’s rank correlation (SRC) test

In SRC test data is analyzed to find out fact that whether male informants have better knowledge than female interviewees or not. SRC is also explores correlation between total number of uses with total number of plants. It was proved that the number of uses of plants also increases as number of plants species increases. It is calculated as:

$$r_{s}\;=\;1-6\left[\frac{\sum d^{2}}{n\left(n^{2}-1\right)}\right]$$

where *d*^2^ the square of the sum of the ranks and n is the number of informants [29].

## Results and discussion

The present ethnobotanical expedition was conducted on mountaineous areas of Dawarian and Ratti Gali (DRG), District Neelam of Azad Jammu and Kashmir, Pakistan in year 2019. EB data generated was compiled in form a checklist of plants, inventory of traditional ethnomedicines and biodiversity conservation status of indigenous plants of DRG areas. The study areas of DRG are hilly terrains with diverse climate and plant vegetation. The area is first time explored using quantitative ethnobotanical approach which resulted many novel data, as no such data is reported in previous literature. This is first document which describes the checklist of wild plants and their ethnobotanical uses are presented in quantitative form which provides clues for future detailed phytochemical and ethnopharmacological research. It was found that indigenous communities of the area generally use plants and their byproducts for different necessities of life.

In the study area (two villages: Dawarian and Rati Gali) a comparison based on six social characters was made prior to plants collection and identification for ethnomedicinal study (Table 1). These characters’ observation directly correlates with plants distribution in the study area. It was observed that more families (52), number of informants (12), average number of families (15–8) and livestock dependence (90%) maximum in Dawarian site as comparison to Rati Gali which is less in all parameters except migration rate (90%) in Ratti Galli, which may be due to severe climatic conditions particularly in chilling snow falling in winter. These findings indicated that less number of plant diversity appeared in Dawarian site as compared with Ratti Galli (where mostly herbs and shrubs were prevalent). The hilly area people of DRG mostly depend on wild and natural resources, particularly on domestic animals for live sustenance. These findings were strongly supported by some ethnobotanist who conducted research on different areas of Azad Jammu and Kashmir [24,28,29].

**Table 1:** Social characteristics of the variable samples between two study sites: Rati Galli and Dawarian of District Neelam of Azad Jammu and Kashmir.

S. No	Social characteristics	Dawarian	Rati Gali
1	Number of families	52	8
2	Number of informants	12	5
3	Reliance on livestock as an income source	90%	30%
4	Average age of informants	70–50	60–30
5	Average number of family members	15–8	10–3
6	Migration ratio	70%	90%

Different geographic characteristics like topography, area climates, population size, altitude or elevation and vegetation size were measured (Table 2). It was determined by the research that landmark diversification of plant species was seen in Dawarian and Rati Gali sites. The phytodiversity variation may be attributed to altitudinal variations such as Dawarian has 1615 meters height with loam rich soil having *Pinus wallichiana* forest. The human population is scattered in diverse area. While Rati Gali is located at 3700 meters having mostly herbs and shrubby vegetation with cool climatic conditions. This climatic, geographic characteristics and elevation differences resulted in plant biodiversity and in Ratti Galli area winter is severe and cold. It is worth to state people from other low land and hot climate areas migrate to these areas during summer for fostering their domestic animals by grazing of lush green grasses and herbs [22].

**Table 2:** Geographical characteristics observation of the two study sites: Rati Galli and Dawarian of District Neelam of Azad Jammu and Kashmir.

S. No.	Sites	Elevation (m)	Geographical characteristics
1	Dawarian	1615	The village has very fertile soil and thick vegetation. Village has ever green thick forest of *Pinus wallichiana*. It is mountainous area. Population of the village is small sized but the area is huge.
2	Rati Gali	3700	This area is located at high altitude. Vegetation mainly consist of herbs or shrubs. There is very low population but area is huge. People migrate here with their domestic animals in summers from different areas.

### Plants collection, identification and preservation

A total of 103 wild indigenous plants (WIPs) were plants were gathered from the selected towns (Dawarian and Ratti Gali) of District Neelam of AJK using standard protocols. The plants were identified using standard protocols as described in above methodology section. The dried and prepared specimens were submitted in Herbarium, Department of Botany voucher numbers for future reference and study. The floristic profile of WIPs was prepared comprising of family name, habit (herb, shrub or tree) and local name of each plant (Table 3). The results depicted that highest number of plants was seen for family Asteraceae (12 species), followed by Lamiaceae (10 spp) and Polygonaceae and Papilionaceae 6 spp each). Similar findings were counted by other taxonomists in other countries where Asteraceae was prevalent and dominant family with its universal distribution [30].

**Table 3:** Familywise Inventory of wild indigenous plants of Dawarian to Ratti Gali, District Neelam of Azad Jammu and Kashmir, Pakistan (note: Herbarium voucher numbers are cited in Table 4).

Sr No	Family	Sr No	Botanical Name of Plant Species	Habit	Local name
1	Asteraceae	1	*Achillea millefolium* L.	Herb	Gandana
		2	*Artemisia japonica* Thunb.	Herb	Chaou
		3	*Anaphalis triplinervis* Clarke	Herb	Butt mehndi
		4	*Artemisia macrophylla* Fisch. Ex Besser	Herb	Chita chaou
		5	*Gerbera gossypina* (Royle) Beauverd	Herb	Kofe
		6	*Ligularia thomsonii* (Clarke) Pojark.	Herb	Jungli surajmukh
		7	*Matricaria chamomilla* L.	Herb	Tamak boti
		8	*Saussurea lappa* (Decne.) Sch.Bip.	Herb	Khut
		9	*Cirsium arvense* (L.) Scop.	Herb	Jungli kandyara
		10	*Sonchus asper* (L.) Hill	Herb	Dhodal
		11	*Senecio chrysanthemoides* DC.	Herb	Chir hand
		12	*Solidago virgaurea* L.	Herb	Pinja phool
2	Amaryllidaceae	13	*Allium griffithianum* Boiss.	Herb	Jungli pyaz
3	Araceae	14	*Arisaema tortuosum* (Wall.) Schott	Herb	Sanp ki boti
4	Aquifoliaceae	15	*Ilex dipyrena* Wall.	Tree	Kandaro
5	Anacardiaceae	16	*Rhus succedanea* L.	Tree	Alkhal
6	Berberidaceae	17	*Berberis 4ustra* Royle	Shrub	Sumbal
		18	*Podophyllum hexandrum* Royle	Shrub	Ban kukri
		19	*Podophyllum emodi* Wall. Ex Hook.f. & Thomson	Shrub	Tra patra
7	Buddlejaceae	20	*Buddleja crispa* Benth.	Shrub	Gansu
8	Buxaceae	21	*Buxus wallichiana* Baill.	Herb	Chiriri
		22	*Sarcococca saligna* Müll.Arg.	Shrub	Shangal
9	Boraginaceae	23	*Cynoglossum lanceolatum* Forssk.	Herb	Chiro
		24	*Onosma bracteata* Wall.	Herb	Gao zuban
10	Betulaceae	25	*Corylus colurna* L.	Tree	Aurni
11	Brassicaceae	26	*Erysimum hieraciifolium* L. f.	Herb	Mirchi
		27	*Erysimum hedgeanum* Al-Shehbaz	Herb	Maneera
12	Convolvulaceae	28	*Convolvulus arvensis* L.	Herb	Berrhi
		29	*Cuscuta reflexa* Roxb.	Herb	Neela tari
13	Campanulaceae	30	*Campanula pallida* Wall.	Herb	Bikh
14	Colchicaceae	31	*Colchicum luteum* Baker	Herb	Sorinjan
15	Celastraceae	32	*Euonymus hemsleyanus* Loes.	Tree	Seeki
16	Crassulaceae	33	*Hylotelephium ewersii* (Ledeb.) H.Ohba	Herb	Loon salooni
17	Cupressaceae	34	*Juniperus communis* L.	Tree	Bentheri
18	Caprifoliaceae	35	*Morina persica* L.	Herb	Bekh-e-Akwar
		36	*Valeriana jatamansi* Jones	Herb	Panchi hola
		37	*Viburnum cotinifolium* D. Don	Shrub	Ukloo
19	Caryophyllaceae	38	*Silene vulgaris* (Moench) Garcke	Herb	Murkun
20	Fumariaceae	39	*Corydalis govaniana* Wall.	Herb	Bhutkas
		40	*Corydalis vaginans* Royle	Herb	Mameri
21	Geraniaceae	41	*Geranium rotundifolium* L.	Herb	Ratan jut
		42	*Geranium villosum* Ten.	Herb	Gull-e-attar
22	Gentianaceae	43	*Swertia paniculata* Wall.	Herb	Charyta
23	Juncaceae	44	*Juncus lacustral* L.	Herb	Jungli ghas
24	Lamiaceae	45	*Ajuga parviflora* Benth.	Herb	Chita chaou
		46	*Ajuga bracteosa* Wall	Herb	Janeadam
		47	*Clinopodium vulgare* L.	Herb	Asaba-el-fetiyal
		48	*Elsholtzia strobilifera* Benth.	Herb	Perilla
		49	*Isodon rugosus* Codd.	Shrub	Pemar
		50	*Mentha longifolia* L.	Herb	Pahari podina
		51	*Origanum vulgare* L.	Herb	Nazbu
		52	*Phlomis bracteosa* Royle.	Shrub	Kukarjari
		53	*Scutellaria linearis* Benth.	Herb	Birch
		54	*Thymus linearis* Benth.	Herb	Ban jamani
25	Oxalidaceae	55	*Oxalis corniculata* L.	Herb	Khatimili
26	Orobanchaceae	56	*Pedicularis brevifolia* D.Don	Herb	Khasturi
27	Orchidaceae	57	*Satyrium nepalense* D.Don	Herb	Gagun
28	Papilionaceae	58	*Astragalus graveolens* Benth.	Herb	Ban phali
		59	*Astragalus heratensis* Bunge	Shrub	Phut Kanda
		60	*Indigofera heterantha* Brandis	Shrub	Kanthi
		61	*Lespedeza juncea* (L.f.) Pers.	Herb	Kanthi ranga
		62	*Vicia sativa* L.	Herb	Chiri panja
		63	*Trifolium repens* L.	Herb	Sinja
29	Pteridaceae	64	*Adiantum aethiopicum* L.	Herb	Kahkawa
		65	*Onychium japonicum* (Thunb.) Kunze	Herb	Kangu
30	Polygonaceae	66	*Aconogonon alpinum* (All.) Schur	Herb	Chikro
		67	*Bistorta amplexicaulis* (D.Don) Greene	Herb	Masloon
		68	*Oxyria digyna* (L.) Hill	Herb	Kakri
		69	*Persicaria mitis* (Schrank) Holub	Herb	Pahari masloon
		70	*Rheum emodi* Wall.	Herb	Chit patra
		71	*Rheum lacustral* D. Don	Herb	Chutyal
31	Polygalaceae	72	*Polygala chinensis* L.	Herb	Sanp ki jari
32	Pinaceae	73	*Abies pindrow* Royle	Tree	Partal
		74	*Cedrus deodara* Don	Tree	Davdaar
		75	*Pinus wallichiana* Jacks.	Tree	Kayal
		76	*Pinus roxburghii* Sarg.	Tree	Cheer
		77	*Picea smithiana* (Wall.) Boiss.	Tree	Kachal
33	Poaceae	78	*Bromus pectinatus* Thunb.	Herb	Pero
		79	*Cenchrus pennisetiformis* Steud.	Herb	Lidder
		80	*Digitaria 6ustral6* (Nees) A.Camus	Herb	Ghaa
		81	*Sorghum halepense* (L.) Pers.	Herb	Baru
34	Primulaceae	82	*Primula 6ustral66e6* Sm.	Herb	Mamera
35	Plantaginaceae	83	*Plantago 6ustral66e* L.	Herb	Kala chamchi part
		84	*Wulfenia amherstiana* Benth.	Herb	**————**
36	Ranunculacea	85	*Actaea spicata* L.	Herb	Moneeri
		86	*Aconitum heterophyllum* Wall. Ex Royle	Herb	Ptrees
		87	*Caltha alba* Cambess.	Herb	Makanpath
37	Rosaceae	88	*Cotoneaster microphyllus* Wall. Ex Lindl.	Herb	Loni
		89	*Rosa microphylla* Roxb. Ex Lindl.	Shrub	Shigari
		90	*Rubus niveus* subsp. *Horsfieldii* (Miq.) Focke	Shrub	Pakana
		91	*Fragaria nubicola* (Lindl.) Lacaita	Herb	Mehwa
38	Rutaceae	92	*Skimmia laureola* Franch.	Shrub	Neri
39	Sapindaceae	93	*Acer cappadocicum* Gled.	Tree	Tera Kanna
		94	*Aesculus indica* Hook.	Tree	Ban khaur
40	Saxifragaceae	95	*Bergenia 6ustral* Sternb.	Herb	Betbewa
41	Sabiaceae	96	*Meliosma simplicifolia* Walp.	Shrub	Bakhaish
42	Salicaceae	97	*Populus alba* L.	Tree	Sufaida
		98	*Salix tetrasperma* Roxb.	Tree	Bheens
43	Symplocaceae	99	*Symplocos paniculata* (Thunb.) Miq.	Shrub	Ludder
44	Taxaceae	100	*Taxus baccata* L.	Tree	Thuni
45	Violaceae	101	*Viola biflora* L.	Herb	Phul naqsh
		102	*Viola canescens* Wall.	Herb	Thandi jari
46	Viscaceae	103	*Viscum album* L.	Shrub	Purakh

### Traditional ethnobotanical data (TEB)

Traditional ethnobotanical (TEB) data of wild indigenous plants (WIPs) was prepared in form of inventory which comprised of botanical name, voucher number, local name, family name, part used, gathering period, mode of use and traditional recipe or uses (Table 4). The results indicated that family Asteraceae showed highest percentage (11.65%), Lamiaceae (8.73%) whereas Polygonaceae (6.79%) species of plant species, respectively. Buxaceae, Boraginaceae, Brassicaceae, Convolvulaceae, Fumariaceae, Geraniaceae, Pteridaceae, Plantaginaceae, Spindaceae, Salicaceae and Violaceae showed 1.94% while Amaryllidaceae, Araceae, Aquifoliaceae, Buddlejaceae, Butelaceae, Campanulaceae, Colchicaceae, Celastraceae, Crassulaceae, Cupressaceae, Caryophyllaceae, Gentianaceae, Juncaceae, Oxalidaceae, Orobanchaceae, Orchidaceae, Primulaceae, Rutaceae, Saxifragaceae, Sabiaceae, Symplocaceae, Taxaceae and Viscaceae 0.97% of plant species being used in different TEB. The family wise inventory with species richness is presented in pie-chart form (Fig 2).

**Fig 2:** Species distribution pattern of each family from Dawarian and Ratti Galli area of Neelam valley of Azad Jammu and Kashmir, Pakistan.

**Table 4:** Traditional ethnobotanical uses of wild indigenous plant species recorded from Dawarian and Ratti Gali, District Neelam Azad Jammu and Kashmir, Pakistan.

S. No	Species name	Family	Collecting Period	Part used	Traditional ethnobotanical uses
1.	*Acer cappadocicum* Gled. MUH-1775	Sapindaceae	Summer	Leaf, Stem, twigs	The gum of tree is used as body tonic. Leaf extract is used for curing of diabetes, dysentery and diarrhea. Leaf and young twigs are used as fodder for animals. Dry wood is used as source of fuel for domestic needs.
2.	*Ajuga bracteosa* Wall. MUH-1776	Lamiaceae	Summer	Root, leaf, flower	Root extract is used for purification of blood. Paste of leaves helpful to cure headache while powder of whole plant is given to treat abdominal pain. The flower powder is used for cure of diabetes. The root tea is used for killing of stomach worms.
3.	*Ajuga parviflora* Benth. MUH-1777	Lamiaceae	Summer	Leaf, root, stem, twigs	The plant leaf extract is used for cure of typhoid and malaria. The root decoction is used for cure of chronic fever and chest pains. It is used as vermifuge. It is used as fodder for domestic goats and animals.
4.	*Allium griffithianum* Boiss. MUH-1778	Amaryllidaceae	Summer	Leaf	The leaf tea or decoction is used to cure fever and cough. It is used as food. It is used as stomach cure and appetizer for easy digestion.
5.	*Aconogonon alpinum* (All.) Schur MUH-1779	Polygonaceae	Summer	Leaf, root	Leaves are used as culinary food. Root is used for the treatment of joints pain. The root powder is used as stomach pain reliever and tonic as wormicidal.
6.	*Actaea spicata* L. MUH-1780	Ranunculaceae	Summer	Root, leaf	Juice of roots is used to kill lice. The leaf extract is used for curing of nerve infirmities, joints inflammation, leucorrhea and rheumatism.
7.	*Aesculus indica* (Wall. Ex Cambess.) Hook. MUH-1781	Spindaceae	Summer	Leaf, root, bark	The leaf decoction is used for cure of skin rashes and irritation. The root powder is used for treatment of rheumatic pains. The bark extract is used for curing of headache. Its leaves are used as fodder. Wood and stem is used as fuel.
8.	*Aconitum heterophyllum* Wall. Ex Royle MUH-1782	Ranunculaceae	Summer	Root, leaf, stem bark	Root’s tea is used for the treatment of fever, vomiting, dysentery, flu cough and abdominal pain with boiled milk. The root decoction is used as expectorant and febrifuge agent. The bark powder is used for cure of inflammation and chronic joints pains.
9.	*Abies pindrow* Royle. MUH-1783	Pinaceae	Summer	Leaf, root	The paste of the leaf is used for curing cuts, wounds and bruises to get rid of bacteria and germs. The root paste is used to cure inflammation of joints. The root tea is used for cure of asthma and cough. Seeds decoction is used for treating fever, hyperglycemia and bronchitis.
10.	*Achillea millefolium* L. MUH-1784	Asteraceae	Summer	Leaf, root	Leaf ash and paste is used for cure bleeding wounds. The leaf decoction is used for dyspepsia and flatulence of stomach. Leaves are chewed to treat teeth pain and gums bleeding. Leaf juice is poured in ear to treat ear pain. Plant root infusion is used to treat T.B., stomach disorder and fever in form of Tea.
11.	*Artemisia japonica* Thunb. MUH-1785	Asteraceae	Summer	Leaf, root, flower	The juice of leaves is used for cough and asthma. The flower decoction is used for cure of vaginitis. The root infusion is used for treating hypertension. The leaf paste is used for cure of joint pains.
12.	*Anaphalis triplinervis* Clarke MUH-1786	Asteraceae	Summer	Leaf, root and stem	The leaf paste is used for cure for wounds and pains of toes. The leaf decoction is used in cure of epilepsy. The whole plant paste is used for treating of animal feet diseases as ethnoveterinary medicines.
13.	*Artemisia macrophylla* Fisch. ex Besser MUH-1787	Asteraceae	Summer	Leaf, shoot, root	Leaves are used for cough and asthma. Shoot is used for fodder. The root decoction is used as relief of edema and diuretic. The leaf cooked as vegetable for cure of constipation. Leaf tea is used as vigour tonic and cure of rheumatic disorders.
14.	*Astragalus graveolens* Benth. MUH-1788	Papilionaceae	Summer	Leaf, Fruit	Leaf is used for cure of wounds. Fruit is eatable and used as antioxidant agent.
15.	*Adiantum aethiopicum* L. MUH-1790	Pteridaceae	Summer	Leaf	Juice of leaves is used for the treatment of chest burning, stomachache and blood purification.
16.	*Arisaema tortuosum* (Wall.) Schott MUH-1791	Araceae	Summer	Leaf, root, tuber	The root decoction is used as wormicide. The extract of leaf is used to cure cattle worms and stomach issues. The dried tubers are used as cure of snake poison.
17.	*Astragalus chlorostachys* Bunge MUH-1792	Papilionaceae	Summer	Leaf	The leaf decoction is used as abortifacient and relief of vaginal pains. The plant is used as fodder for the livestock and cattle.
18.	*Bergenia locustral* (Haw.) Sternb. MUH-1793	Saxifragaceae	Summer	Leaf, root	Extract of leaf is used for cure of earaches. The root decoction is used as a tonic in treatment of fevers, diarrhoea and pulmonary affections.
19.	*Bromus pectinatus* Thunb. MUH-1794	Poaceae	Summer	Leaf, whole plan	It is used as fodder with increasing of milk yield in cattle. The plant is also used as fuel agent in dried form.
20.	*Berberis 10ustra* Royle MUH-1795	Berberidaceae	Summer	Leaf, root	Dried leaves powder is used for the treatment of headache, stomachache. The root decoction is used for cure of joints pain and toothache. Boiled water of roots is used to treat internal wounds, especially bone fracture.
21.	*Bistorta amplexicaulis* (D.Don) Greene MUH-1796	Polygonaceae	Summer	Root, Leaf	Dried root is used as tea to cure stomachache. The herbaceous roots are tonic for enhancing of cow milk. The root decoction is used for cure of toothache. The whole plant is also used as fodder or cattle. Root paste is used as cure of snake poison.
22.	*Buddleja crispa* Benth. MUH-1797	Buddlejaceae	Summer	Root, leaf	The root infusion is used for curing wound healing by increasing platelets. Its leaf extract is used for inflammation and analgesic purpose. It is used as fodder for indigenous pets and cattle.
23.	*Buxus wallichiana* Baill. MUH-1798	Buxaceae	Summer	Leaf, root, seed	Dried leaves are used in the treatment of joints pain and muscles pain. The root decoction is used for cure of syphilis. The seed powder is used as purgative agent.
24.	*Convolvulus arvensis* L. MUH-1799	Convolvulaceae	Summer	Leaf, stem, root	Leaf is used as vegetable which is purgative and laxative. The stem paste is used for treating of joints pain. It is also used as fodder.
25.	*Cirsium arvense* (L.) Scop. MUH-1800	Asteraceae	Summer	Leaf, root, stem	The leaf decoction is used for cure of edema. The root powder is used for cure of hepatic issues. Powdered form mix with water is used as tonic.
26.	*Campanula pallida* Wall. MUH-1801	Campanulaceae	Summer	Leaf, stem, root	The leaf is used to cure bactericidal and fungicidal. The root decoction is used for treating scabies. The leaf and stem is used as fodder.
27.	*Cynoglossum lanceolatum* Forssk. MUH-1802	Boraginaceae	Summer	Leaf, root	The foliar past is applied on abscess to remove pus. It is also use in asthma. The leaf decoction is used for cure of eye ailments. The root infusion is used for cure of chest infection and bronchitis.
28.	*Cuscuta reflexa* Roxb. MUH-1803	Convolvulaceae	Summer	Whole plant, stem	Juice of the whole plant used to increase the length of hairs and make strong. It is also used as fodder. Its decoction is used in jaundice and cure of spleen disorders. The infusion is used for treating urinary issues. The powder mixed with desi ghee/butter is used for cure of weak muscles and their pains.
29.	*Cedrus deodara* (Roxb. Ex D.Don) G.Don MUH-1804	Pinaceae	Summer	Leaf, stem, fruit, root, wood	The leaf decoction is used for treating of piles. The root burnt used to cure epilepsy. The fruit is used for renal infection and fever. The stem bark is used for curing urinary bladder issues. Oil of wood is used for toothache, applied to skin for skin problems. Wood is also used as fuel.
30.	*Colchicum luteum* Baker MUH-1805	Colchicaceae	Summer	Leaf, root, stem, flower	Juice of plant is used for purification of blood. The leaf decoction is used for curing gout and joint pain. The root infusion is used for cure of liver disorders and enlarged spleen.
31.	*Corylus colurna* L. MUH-1806	Butalaceae	Summer	Fruit, leaf	Fruit is eatable is used as vigour. The leaf extract is used as antioxidant. Leaf extract is useful as cure of snake poison.
32.	*Corydalis vaginans* Royle MUH-1807	Fumariaceae	Summer	Sap, root	The sap of the plant is used in the treatment of eye diseases. The root decoction is used to cure epilepsy.
33.	*Cotoneaster microphyllus* Wall. Ex Lindl. MUH-1808	Rosaceae	Summer	Leaf, root, stem	The leaf decoction is used for treating of diarrhoea. The root powder is used as effective to cure wounds. The leaf and stem is used as fodder for cattle and goats.
34.	*Corydalis govaniana* Wall. MUH-1809	Fumariaceae	Summer	Leaf	The juice of leaf is used for the treatment of fever and skin problem.
35.	*Caltha alba* Cambess. MUH-1810	Ranunculaceae	Summer	Leaf, whole powder	The dried powder or juice of this plant is used to reduce muscle pain and sedative.
36.	*Cenchrus pennisetiformis* Steud. MUH-1811	Poaceae	Summer	Leaf, stem	The leaf extract is used for cure of bacterial infections. The stem and leaf parts are used as fodder for cattle and rodents.
37.	*Clinopodium vulgare* L. MUH-1812	Lamiaceae	Summer	Leaf	A sweet and aromatic herb tea is made from the fresh leaf for cure of headache and migraine pain.
38.	*Digitaria cruciata* (Nees) A.Camus MUH-1813	Poaceae	Summer	Seed, leaf, root	The seed powder or flour is used as tonic for body vigour. The root decoction is used for curing of stomach disorders. The leaf extract is used as bioherbicidal. It is used as fodder for cattle and goats.
39.	*Erysimum hieraciifolium* L. f. MUH-1814	Brassicaceae	Summer	Leaf, root, whole plant	The leaf decoction is used for cure of foot rot. The root infusion is used for treatment of pimples and bruises on legs. The whole plant is used as food and source of vegetable.
40.	*Erysimum hedgeanum* Al-Shehbaz MUH-1815	Brassicaceae	Summer	Leaf, whole plant	This is poisonous herb. The juice of whole plant is use to kill lices in animals.
41.	*Euonymus hemsleyanus* Loes. MUH-1816	Celastraceae	Summer	Leaf, root, whole plant	The leaf decoction is used as tonic for hair growth. It is used as fodder cattle and rodents.
42.	*Elsholtzia strobilifera* (Benth.) Benth. MUH-1817	Lamiaceae	Summer	Leaf, root, stem	The leaf tea is useful for cure of cold and flu. The root infusion is used for treating indigestion, flatulence and diarrhea. The stem bark is used for cure of pharyngitis disorders. The whole plant is used as fodder cattle and rodents.
43.	*Fragaria nubicola* Lacaita MUH-1818	Rosaceae	Summer	Fruit, leaf	Fruit is eatable and used as antioxidant agent. The leaf decoction is used for curing of blemishes infirmities. The fruit extract with milk is used for damaged and broken nerve disorders. The leaf smoke is used for treating of lungs issues.
44.	*Geranium rotundifolium* L. MUH-1819	Geraniaceae	Summer	Root, Leaves	Dried root powder is doted on wounds. The dried roots were grinded, sugar and milk are added in it, and then used for pain relief of joints. The root decoction is used to cure epilepsy.
45.	*Geranium villosum* Ten. MUH-1820	Geraniaceae	Summer	Leaf, bark and whole plant	It is used as food for cure of edema. The leaf and bark paste is used for broken and fractured legs and joints.
46.	*Gerbera gossypina* (Royle) Beauverd MUH-1821	Asteraceae	Summer	Leaf, root, stem	The leaf decoction is used cure of hair disorders. The root powder is used for treating the rashes and foot allergy. It is used as fodder cattle and rodents.
47.	*Hylotelephium ewersii* (Ledeb.) H.Ohba MUH-1822	Crassulaceae	Summer	Leaf	It is believed to be having cooling effect if the juice of the leaves mix with water and drink.
48.	*Ilex dipyrena* Wall. MUH-1823	Aquifoliaceae	Summer	Leaf, stem	It is used as fodder. It is also the source of fuel and wood.
49.	*Indigofera heterantha* Brandis MUH-1824	Papilionaceae	Summer	Leaf, Shoot	The leaf decoction is used for cure of stomach disorder and abdominal pains. Shoots are used as fodder, branches as ropes, brooms and fuel.
50.	*Isodon rugosus* (Wall.) Codd MUH-1825	Lamiaceae	Summer	Leaf, root	Juice of the leaves is used for stomachache. The root decoction is used for respiratory and cardiovascular problems.
51.	*Juncus arcuatus* Wahlenb. MUH-1826	Juncaceae	Summer	Whole plant	It is used as fodder cattle and rodents. It is used as fuel in dried form.
52.	*Juniperus communis* Brand. MUH-1827	Cupressaceae	Summer	Wood, leaf, root	The decoction of root is used for cure of inflammation and diarrhea. The leaf extract is used as microbicide and antiseptic. It is the source of fuel and commercial wood.
53.	*Lespedeza juncea* (L.f.) Pers. MUH-1828	Papilionaceae	Summer	Leaf, root	The decoction of root is used as cure of diarrhea and dysentery. The leaf tea is used for stomach pains. It is used as fodder cattle and rodents.
54.	*Ligularia thomsonii* Clarke. MUH-1829	Asteraceae	Summer	Root, leaf	Dried root or powdered of root is used in the treatment of asthma. The leaf infusion and salad is stimulator of blood flow, reduce inflammation and stopping cough.
55.	*Mentha longifolia* L. MUH-1830	Lamiaceae	Summer	Leaf, shoot.	Shoot extract is used for stomachache and gas trouble. Juice of leaves expels worms from the stomach. It is also as condiment. The root decoction is used to cure cardiovascular disorders.
56.	*Matricaria chamomilla* L. MUH-1831	Asteraceae	Summer	Root, leaf, stem bark	Root powder is used for toothache. The leaf decoction is used in relief of fever and inflammation. The bark is used for cure of menstrual cycle regulator.
57.	*Morina persica* L. MUH-1832	Caprifoliaceae	Summer	Aerial parts	It is used for treatment of cold. Its leaf extract is used as bactericidal and fungicidal herbal medicine.
58.	*Meliosma simplicifolia* (Roxb.) Walp. MUH-1833	Sabiaceae	Summer	Leaf, Wood	Leaf decoction is used as cure of inflammation reducer of legs and broken joints. The leaf is used as fodder. Its wood is source of fuel.
59.	*Oxalis corniculata* L. MUH-1834	Oxalidaceae	Summer	Leaf, Flowers	Juice of leaves and flowers mixed together is used for the treatment of eyes.
60.	*Onychium japonicum* (Thunb.) Kunze MUH-1835	Pteridaceae	Summer	Leaf, root	Leaf is used as vegetable for laxative purpose. Dried root or powdered root is used for the treatment of asthma and flu.
61.	*Oxyria digyna* (L.) Hill MUH-1836	Polygonaceae	Summer	Shoot, root, leaf	Shoot extracts are used for constipation, liver disorders and stomachache. Root decoction is used for cure of stomachache.
62.	*Onosma bracteata* Wall. MUH-1837	Boraginaceae	Summer	Root, leaf	Powder of dry root is used against asthma and bronchitis. Decoction of leaf is given in stomach and bladder irritation.
63.	*Origanum vulgare* L. MUH-1838	Lamiaceae	Summer	Leaf, root	The leaf poultice is used for muscles pain and broken bones. The root tea is used for cold cure and toothache. It is also as vegetable and fodder.
64.	*Polygala chinensis* L. MUH-1839	Polygalaceae	Summer	Leaf, root, stem	This root powder plant is used for treatment of snake bites. The leaf extract is used as fever cure and expectorant for cough and bronchitis. The leaf extract is also used to cure cardiovascular disorders.
65.	*Phlomis bracteosa* Royle ex Benth. MUH-1840	Lamiaceae	Summer	Leaf, Flower	Leaf powder is mixed in tea and used against cough and cold. Flowers are crushed and used against toothache.
66.	*Pedicularis brevifolia* D.Don MUH-1841	Orobanchaceae	Summer	Leaf, Root	Leaf decoction is used for the treatment of cough, fever and asthma. The leaf poultice is used for allergy and skin disease. Dried or powdered root is used for the treatment of stomachache.
67.	*Primula lacustra* Sm. MUH-1842	Primalaceae	Summer	Stem, leaf	Juice of stem is used for eye diseases. Leaf extract is used for cure of scabies.
68.	*Podophyllum hexandrum* Royle MUH-1843	Barberidaceae	Summer	Leaf, root	Leaf powder is used in the treatment of asthma. Root is used to reduce goiter and other sore throat infections.
69.	*Populus alba* L. MUH-1844	Salicaceae	Summer	Leaf, root, bark	The leaf decoction is used to cure gout, joint pain and arthritis. The root infusion is used for backbone and lumber pains. The stem bark is used as cure of liver inflammation and debility issues. Leaf are used as fodder. Wood is used as fuel.
70.	*Plantago lanceolata* L. MUH-1845	Plantaginaceae	Summer	Leaf, root, stem bark	The leaf decoction is used as laxative. The root tea is used for cure of cold, flu and fever. The bark extract is employed is used for cure of debility and body general weakness.
71.	*Persicaria mitis* (Schrank) Holub MUH-1846	Polygonaceae	Summer	Root, leaf	Tea is made by root which help to reduce the joints pain. Leaf is used for cure of stomach pains.
72.	*Picea smithiana* (Wall.) Boiss. MUH-1847	Pinaceae	Summer	Leaf, root, wood	The leaf extract is used for cure of wounds and chilling pains. The root decoction is used for treating the stomachache. Wood is the source of fuel.
73.	*Podophyllum emodi* Wall. Ex Hook.f. & Thomson MUH-1848	Berberidaceae	Summer	Leaf, root, stem bark	The leaf decoction is used to cure constipation and burning sensation. The root tea is used to cure colds, fever and cough. The bark powder is used for cure of wounds. It is used as fodder cattle and rodents.
74.	*Pinus wallichiana* A.B.Jacks. MUH-1849	Pinaceae	Summer	Leaf, stem bark, root, resin, seeds	The smell of resin reduce severe cough. Leaf decoction is used cure heat of stomach and chest infection. The infusion of bark is used for cure of dysentery. Wood is used to make house thatching and source of fuel as well. Cones are used for fuel purposes and seeds are edible as nuts. The resin is used to make coal for paving roads.
75.	*Pinus roxburghii* Sarg. MUH-1850	Pinaceae	Summer	Resin, leaf, bark and flower cone	The extract of leaf is used to kill worms and used as septic agent. The infusion of bark is used for dysentery and heat or burning sensation of feet. Wood is used for furniture and fire purpose. Smoke is used to repel the mosquitoes and other insects. Flower extract is also used to cure cardiovascular disorders.
76.	*Rosa macrophylla* Lindl. MUH-1851	Rosaceae	Summer	Fruit, root, flower	Fruit is used in fever to cure from it. The root powder is used for cure of brunt wounds. The flower is used to make admixture of flower with sugar and is used for cure of body tonic.
77.	*Rheum emodi* Wall. MUH-1852	Polygonaceae	Summer	Leaf, root, stem bark	The leaf extract is used as laxative and urination. The root infusion is used for cure of fever and cough. The stem bark decoction is used for treating of menstrual or other sexual disorders.
78.	*Rubus niveus* subsp. *Horsfieldii* (Miq.) Focke MUH-1853	Rosaceae	Summer	Fruit, root and leaf	Fruit is eatable and used as tonic of body. The leaf decoction is used for cure of debility and menstrual disorders. The root extract is used to treat eye problems.
79.	*Rheum lacustral* D. Don MUH-1854	Polygonaceae	Summer	Root, Leaf	Leaf decoction is used to cure stomachache and it is cooked as vegetable which is laxative and used to cure constipation. Paste of root is used for wound healing.
80.	*Rhus succedanea* L. MUH-1855	Anacardiaceae	Summer	Leaf, root, stem	The root extract is used as antidote for scorpion sting. The root infusion is applied for as febrifuge and antivinous. The stem bark is used for cure of ophthalmic disorders. It is used as fodder. It is also source of fuel. Stem bark decoction is used to cure kidney disorders.
81.	*Saussurea lappa* (Decne.) Sch.Bip. MUH-1856	Asteraceae	Summer	Root, leaf	Powder of root is used for cough and toothache. The extract of root is used as vermifuge for intestinal worm. Juice of root is used to cure rheumatism and pneumonia. Its root is used for cure of tuberculosis and epilepsy.
82.	*Silene vulgaris* Garcke. MUH-1857	Caryophyllaceae	Summer	Leaf, whole plant	It is used as vegetable laxative. The plant has many nutritive worth. It is also used for fodder for rodents in local area.
83.	*Sonchus asper* Hill. MUH-1858	Asteraceae	Summer	Leaf and whole plant	Its leaf decoction is used for cure of bleedings. It is known as best antioxidant for cure of different infirmities. Fresh leaves and stem is cooked as vegetable. It is used as fodder as well.
84.	*Sorghum halepense* Pers. MUH-1859	Poaceae	Summer	Seed, leaf, stem, root	Seed flour is used as body tonic. Juice of root is used for the asthma. Leaf decoction is used for urinary irritation. It is also used for fodder.
85.	*Senecio chrysanthemoides* DC. MUH-1860	Asteraceae	Summer	Leaf, root, whole plant	Leaf decoction is used for cure of rashes and bruises. Root paste us used for scorpion sting antidote. It is used as vegetable.
86.	*Skimmia laureola* Franch. MUH-1861	Rutaceae	Summer	Leaf, root, stem wood	Tea is made by dry leaves which is very effective in joints pain, muscles pain, stomach pain and bone pain. Powdered root also used in deserts.
87.	*Salix tetrasperma* Roxb. MUH-1862	Salicaceae	Summer	Leaf, shoot, whole plant	Leaf infusion is used as bactericidal. It is used antidiabetic tonic. It is used as fodder. Wood is used as fuel. Shoot extract is also used to cure cardiovascular disorders.
88.	*Symplocos paniculata* (Thunb.) Miq. MUH-1863	Symplocaceae	Summer	Leaf, root	Powdered leaf is used with cow milk is used for treatment of menorrhagia. The leaf extract is applied on eye disease like irritation. Its root decoction is used for cure of dysentery.
89.	*Sarcococca saligna* Müll.Arg. MUH-1864	Buxaceae	Summer	Leaf, root	Tea of leaf is used in constipation, blood purification and muscles relaxation. The root powder with hot milk or water is used as laxative. The root decoction is used for cure of muscular pains and blood cleanser in the study area.
90.	*Satyrium nepalense* D.Don MUH-1865	Orchidaceae	Summer	Tuber, leaf	Tubers are used as tonic and to cure dysentery and malaria fever. The leaf and tuber tea is used for cure of backbone pain. Its decoction is used for curing nephritis and kidney disorders. The leaf paste is used for cure of erectile dysfunction.
91.	*Scutellaria linearis* Benth. MUH-1866	Lamiaceae	Summer	Leaf, root	Leaf powder is used to reduce inflammation and diarrhea. The root decoction is used for treatment of analgesic problems. The plant is used for antinociceptive agent in different drug preparation. It is neuro-stimulus booster.
92.	*Swertia paniculata* Wall. MUH-1867	Gentianaceae	Summer	Leaf, root	Leaf extract is used to cure hepatic disorders. The root decoction is used to treat diabetes. Powdered plant is used to cure from fever.
93.	*Solidago lacustralis* Fisch. Ex Herder MUH-1868	Asteraceae	Summer	Leaf, shoot, root	Leaf paste is used to cure of burns. Root powdered plant is used to heal wounds and cure of pus and pain. It is used as cure of edema by release of excessive water. Root decoction us used to cure kidney stones.
94.	*Thymus linearis* Benth. MUH-1869	Lamiaceae	Summer	Leaf, root, whole plant	Tea is made by this plant which help to reduce fats in body, abdominal pain and gas trouble.
95.	*Taxus baccata* L. MUH-1870	Taxaceae	Summer	Leaf, root, wood	The leaf extract is used to treat cold and fever. The root powder is used for treatment of cough and chest pains. It is also used for preparation of taxol medicines. The plant is used for source of fuel.
96.	*Trifolium repens* L. MUH-1871	Papilionaceae	Summer	Leaf, root, stem	Leaf extract is used to cure eye diseases. The root decoction is used to treat col and fevers. The stem bark is used to cure leucorrhea. This whole plant is used as vegetable
97.	*Viola biflora* L. MUH-1872	Violaceae	Summer	Leaf, flower	Leaf tea is used to cure flu and colds. The decoction is used for chest infections and cure of soar throat. Flower tea helps in cough headache and flu.
98.	*Vicia sativa* L. MUH-1873	Papilionaceae	Summer	Leaf, seed	Leaf is cooked and used vegetable. The leaf decoction is used to treat Parkinson disease. Seeds infusion is used as cure depressant and hypertension.
99.	*Viburnum cotinifolium* Don. MUH-1874	Caprifoliaceae	Summer	Fruit, leaf, root	Fruit is eatable and used as blood purifier. Leaf extract is known for cure of menorrhagia. The bark is used to muscular pains and cramps. The root tea or infusion is used as laxative to cure constipation.
100.	*Viscum album* L. MUH-1875	Viscaceae	Summer	Leaf, seed, root, bark	Leaf extract is used in the treatment of cough and asthma. Root powder is used to cure nervousness and fatigue issues. The seed roasted and taken with milk to cure insomnia and lesser immunity. The bark of stem is used to cure panic attacks and mental agitation. The root decoction is used to cure cancer and joint pains. The tea of leaf is used for cure of hypertension.
101.	*Viola canescens* Wall. MUH-1877	Violaceae	Summer	Leaf, root, flower	Leaf powder is used for cure of cough and flow. Tea of flowers is given internally in the treatment of coughs and asthma. The flower decoction is also used in cure of cancer disease. The tea of viola is useful in cure of malaria and immunity development.
102.	*Wulfenia amherstiana* Benth. MUH-1878	Plantaginaceae	Summer	Whole plant, root	Root decoction us used to cure kidney disorders. It is used as fodder cattle and rodents.
103.	*Withania coolgulans* L. MUH-1879	Solanaceae	Spring	Leaf, seed	The leaf decoction is used to cure fatigue, disability. The seed powder is used for cure of insomnia. The seeds in fat/desi ghee is used for body impotence and nervous activeness.

In this exploration, TEB uses of 103 plant species belonging to 46 families were recorded and presented in alphabetical order. Asteraceae was the dominant family of study area with 12 plant species. The leaf decoction of *Artemisia macrophylla* Fisch ex. Besser is used to cure of cough and asthma. The leaf extract or juice of *Artemisia japonica* Thunb is used for whooping cough and asthma disorders. The similar ethnomedicinal study had reported in past on different areas of Azad Jammu and Kashmir, Pakistan where similar uses are cited [13,26–28].

The present study revealed that 78 species (75%) had single ethnobotanical use, 21 species (20%) had dual use and four species (3%) had multiple uses. The plants have been used in different categories such as food, medicines, fruits, vegetables, timber wood, fodder, shelter or house construction and fuel source (Table 4). Similar ethnobotanical studies were conducted on the plants of District Kotli and District Bhimber of Azad Jammu and Kashmir, Pakistan [6,26–28]. In which it was investigated that 93 plant species of 46 families had different form of uses i.e. 52.68% plants were known for single usage, 37.63% plants had dual use, 7.52% for triple usage and 2.15% plants taxa were known for multiple ethnobotanical uses. It was proved that rural people primarily depend on wild indigenous plants for food, fodder and medicines to cope their life necessities. Some of WIPs have also been reported as ethnoveterinary medicines (EVMs). Similar findings have been reported in other ethnobotanical studies in different areas of Khyber Pakhtunkhwa province of Pakistan [31].

### Summary of ethnobotanical investigation

To summarize ethnobotanical data, on the basis of single or more recipe uses, all 103 plants species were categorized into four types. The data is presented in four types with 75.72% plants were being used in single recipes, 20.38% were used in dual usages (in admixture form) and 3.88% plants had been reported having multiple usages. A pictorial form data is shown in pie-chart shape (Fig 3).

**Fig 3:** Graphical presentation of plants on the basis of their usage from study area of Dawarian and Rati Gali, District Neelam of Azad Jammu and Kashmir, Pakistan.

### Single-usage plants

The study revealed that out of 103 plants, about 78 plants were having their single form recipe being used to cure different infirmities by the local communities. Out of 78 plants, medicinal plants were 45 (57.69%), whereas food, fodder and fuel were 15 (19.23%), 15 (19.23%) and 3 (3.84%), respectively. A pie-chart of all single-usage plants is given in Fig 4. It is believed that either these single use-plants have very high medicine potential so individually used for cure of different ailments or these are easy to collect and cheap. So, indigenous population prefer to use this recipe form using different modes of recipe preparation i.e. decoction, powder, infusion, extract, paste etc. These findings (single-use recipes of each plant) were strongly correlated with Uniyal medicinal practices in Kangra district of Himachal Pradesh, Western Himalaya [32].

**Fig 4:** A pie-chart of single-usage on the basis of their usage from study area of Dawarian and Rati Gali, District Neelam of Azad Jammu and Kashmir, Pakistan.

### Dual-usage plants

The plants that are used for two key purposes are called dual-usage plants. For example, *Artemisia macrophylla* is used for medicinal as well as fodder. Out of 103 plants species, 21 (20.38%) were representing dual-usage plants. There were six categories of dual-usage of plants representing 21 species, i.e. medicinal & food and fodder & fuel were 7 (33.33%) while medicinal & fodder and food & fodder were 3 (14.28%) and 2 (9.52%), respectively. Medicinal & condiments and medicinal & fuel were 1 (4.76%). A pie-chart of all dual-usage plants is given in (Fig 5). Many researchers positively correlate with our findings as Polat and his co-researchers discussed an ethnobotanical use of medicinal plants in Espiye and its surroundings in 2015 which had dual uses in many areas of research [33].

**Fig 5:** A pie-chart of dual usage plants the basis of their usage from study area of Dawarian and Rati Gali, District Neelam of Azad Jammu and Kashmir, Pakistan.

### Multiple-usage plants

The plants which are used for multiple purposes are called multiple-usage, e.g. *Pinus wallichiana* Jacks. Is used for fuel, furniture, medicinal and thatching. Out of 103 plant species, four were representing multi-usage plants category. There were three categories of multi- usage plants representing four plant species. Out of four plants, fodder, ropes and fuel were 1(25%), medicinal, furniture, fuel and thatching were 2(50%) while Medicinal, food and fodder were 1(25%). A list of all the multiple-usage plants, their local names and families is given in (Table 6). While a pie-chart of all multiple-usage plants is given in (Fig 6). Similar multiple Traditional use of medicinal plants among Kalasha, Ismaeli and Sunni groups in Chitral District, Khyber Pakhtunkhwa province Pakistan were documented in year 2016. These multiple uses of any plant proves that the plants have very high medicinal and domestic value in life of indigenous communities. It also proves that these plants are facing severe biotic threats being exploited by the local and national markets for domestic and commercial purposes [31–35].

**Fig 6:** A pie chart of multiple-usage plants the basis of their usage from study area of Dawarian and Rati Gali, District Neelam of Azad Jammu and Kashmir, Pakistan.

One similar research was conducted on the plants of Darguti area of Tehsil Khuiratta where plants multiple uses being employed by the local population of AJK (Pakistan) while similar type of research works have also been cited in other parts of world where it is proved that high number of plants possess very significant worth from this district which falls in subtropical region [16,36–40] while the reported study area occurs in temperate region [41,42], hence only few plants species were used in multiple use form that may be rich diversity of plants present in the area and people have enough choice to use various available to cope their life necessities.

The medicinal dosage forms preferably used by the study area people include: infusion, juice, powder, paste, extract, tea, decoction and oil for the treatment of different diseases. It is concluded that decoction is the very common form of dosage (20%), followed by powder (17%), extract (14%), tea (13%), paste (9%), juice (7%), chewing (4%) and oil (3%) is least used form (Fig 7) being used by the indigenous communities. It is due to easy preparation of powder or pills from plants parts which have long shelf life and easy to eat or engulf. The other form decoction and extract are popular in use because they have high efficacy for cure of different infirmities in the local areas of AJK and Pakistan. Similar results have been reported in the past research workers that decoction, powder and extract are prevalent form of recipe use-form in different areas of world [24,26].

**Fig 7:** Depicting recipe forms used for the treatment of different diseases in study area of Dawarian and Rati Gali of District Neelam of Azad Jammu and Kashmir.

For ethnobotanical (EB) purpose-uses of wild indigenous plants (WIPs) are fodder, food, fuel, hedging, thatching, shadow, shelter and construction were used by local people. Among these EB uses highest percentage (37%) is used as fodder, food (32%), fuel 17%, furniture and construction (6%) each. Similar studies were conducted on the plants of Kel village of Neelum Valley, Azad Jammu and Kashmir. They investigated 50 plants belonging to 33 families from the study area where plants have been used in form of food, fodder, shelter, forage and fuel [24,26–28]. The most common part of plant being used for ethnomedicines or EB uses was leaf (18%), followed by seed (17%), root (13%), shoot and bud (9%) each, tuber (7%), bark (6%), sap (5%), and resin is 4% (Fig 8). The highest percentage of leaf used in ethnomedicines or in ethnobotanical uses because these have high conc. of phytoconstituents because of its active photosynthesis machinery process. These are also regenerated as new leaf shape due to primary and secondary growth phenomena. Seeds are easy to collect, long storage time and their accessible availability around the year make them 2^nd^ higher use part of plant (Fig 9). Similar reasons and reports have been cited in the previous research works [27,34].

**Fig 8:** Different parts of plants used for the treatment of different diseases in study area of Dawarian and Rati Gali of District Neelam of Azad Jammu and Kashmir.

**Fig 9:** Different ethnobotanical uses of plants used by local people in different categories in study area of Dawarian and Rati Gali of District Neelam of Azad Jammu and Kashmir.

### Statistical analysis

In the study different quantitative ethnobotanical analysis tools were applied to verify the authenticity of data collected from indigenous people. One commonly used tool is fidelity level (FL) which was employed on the data which depicted that *Allium griffithianum* (Jungli pyaz) and *Fragaria nubicola* (Mehwa) are leading species with 75% use-value which is frequently used by local people of Dawarian for treatment of cure of fever & cough and broken nerve disorders, respectively. Second highest FL 72% for *Mentha longifolia* (Pahari podina) which is used for stomachache, flatulence and condiments. The leaf paste of *Abies pindrow* (Partel) is applied on cuts and wounds bruises to get rid of bacteria and germs. Its wood is also the source of fuel. The results of research are coincident with work of Ahmad and his colleagues who conducted similar studies on the plants of Kel village, Neelum Valley, Azad Jammu and Kashmir [24]. They described that highest FL (95%) was for *Berberis lyceum* being utilized in jaundice, hepatitis, typhoid, fever and tuberculosis issues. In that it was found that *Dioscorea bulbifera*, *Impatiens glandulifera* (90%) were utilized in stiffness, joint torment and *Artemisia vulgaris* (90%) was utilized in liver issues. Additionally, FL level was likewise applied by Farooq in an exploration bunch where similar findings were determined [26]. In our research work, five plant species including *Berberis lyceum* (FL = 97.78%), *Isodon rugosus* (FL = 95.71%), *Saussurea lappa* (FL = 94.74%), *Aconitum heterophyllum* (FL = 92.71%) and *Taxus baccata* (91.58%) had shown very good fidelity level which confirmed that these plants have high medicinal worth in study area (Table 5). Many of these like *Saussurea lappa*, *Aconitum heterophyllum* and *Taxus baccata* are collected from wild and sold on commercial scale to local and national markets for drug development. *Taxus baccata* is used for production of cancer and tumor treatment disease. Similar findings have been reported in other parts of AJK and Pakistan in various ethnobotanical research works indicating that local people of rural and mountains areas still rely on plant for different needs of life [43–48].

**Table 5:** Fidelity level of plants in study area of two villages Dawarian and Ratti Gali of AJK, Pakistan.

Sr.No	Species name	Local name	NP	N	FL
1.	*Acer cappadocicum*	Tra kanna	45	70	64.29
2.	*Ajua bracteosa*	Jan-e-Adam	56	85	65.88
3.	*Ajuga parviflora*	Chita chaou	51	74	68.92
4.	*Allium griffithianum*	Jungli pyaz	32	55	58.18
5.	*Aconogonon alpinum*	Chikro	57	90	63.33
6.	*Actaea spicata*	Moneeri	66	87	75.86
7.	*Aconitum heterophyllum*	Ptrees	89	96	92.71
8.	*Abies pindrow*	Partal	45	60	75.00
9.	*Artemisia macrophylla*	Chita chaou	23	45	51.11
10.	*Astragalus graveolens*	Ban phali	45	75	60.00
11.	*Adiantum aethiopicum*	Kahkawa	21	35	60.00
12.	*Berberis lycium*	Sumbal	88	90	97.78
13.	*Fragaria nubicola*	Mehwa	45	55	81.82
14.	*Isodon rugosus*	Pemar	67	70	95.71
15.	*Mentha longifolia*	Pahari podina	66	75	88.00
16.	*Plantago lanceolata*	Kala chamchi part	71	79	89.87
17.	*Rosa macrophylla*	Shigari	44	75	58.67
18.	*Saussurea lappa*	Kuth	90	95	94.74
19.	*Silene vulgaris*	Murkun	35	45	77.78
20.	*Sonchus asper*	Dhodal	44	50	88.00
21.	*Thymus linearis*	Ban jamani	72	85	84.71
22.	*Taxus baccata*	Thuni	87	95	91.58
23.	*Trifolium repens*	Sinja	55	70	78.57
24.	*Viola biflora*	Phul naqsh	78	90	86.67
25.	*Vicia sativa*	Chiri pancha	54	75	72.00
26.	*Viburnum cotinifolium*	Ukloo	58	70	82.86
27.	*Viscum album*	Purokh	68	80	85.00
28.	*Valeriana jatamansi*	Panchi hola	61	85	71.76
29.	*Viola canescens*	Thandi jari	31	35	88.57

In another parameter family index (FI) was determined according to number of plants used in different ethnobotanical perspectives in the study area. FI results indicated that family Asteraceae ranked 1^st^ with 12 species, followed by Lamiaceae (10 spp.) and lowest FI was 04 species for Rosaceae (Table 6). This high occurrence of plants of Asteraceae is that plants of this family are cosmopolitan and have wide of range of occurrence, probably due to good seed dispersal mechanism. These findings were very closely supported by Mehwish and her colleagues who stated that Asteraceae has high occurrence in AJK areas [28,30]. FL and FI both along with other statistical analytical tools have been employed in different research studies which proves the efficacy of medicinal plants being used as herbal therapeutics and also production of allopathic medicines using different pharmaceutical procedures in the industries [49–51].

**Table 6:** Family index in study area of two villages Dawarian and Ratti Gali of AJK, Pakistan.

S. No.	Family	Number of species	Ranking
1	Asteraceae	12	1^st^
2	Lamiaceae	10	2^nd^
3	Polygonaceae	7	3^rd^
4	Papilionaceae	6	4^th^
5	Pinaceae	5	5^th^
6	Poaceae	4	6^th^
7	Rosaceae	4	7^th^

Another statistical tool, Spearman’s rank correlation (SRC) test was employed for authentication of ethnomedicinal uses of the wild indigenous plants (WIPs) of Dawarian and Ratti Gali of District Neelam of AJK. SRC is used to confirm that (i) “*either the number of uses of plants increases with increases in the number of species*?” and (ii) *to correlate traditional indigenous knowledge (TIK) of males and females to find out facts that either females have better TIK as compared to males or not*”. It was proved that number of ethnomedicinal uses increases with increases the number of plant species in the study. Furthermore it was confirmed that old village women had more TIK of wild plants and this may be due to fact that female mostly live in their native towns and have more knowledge of herbal therapeutics as compared to men who mostly go abroad or out of hometowns for jobs and other purposes, so they forget or have less opportunities for using and dependency on WIPs to cure various infirmities (Tables 10 and 11). Where s*R* values for male were 0.733 while for female s*R* was0.893. Both readings are near to p = 1; which proves that indigenous population (male and female) prevalently depend on wild resources for cure of different infirmities (Table 7). But female population had more knowledge and dependence than male in the area. Similar studies were conducted by Ahmad and his colleagues [24] in Kel area of Neelum Valley of Azad Jammu and Kashmir where he said female population had more information of plants for different domestic and commercial uses as compared to men (Table 8). In other study, Amjad and his colleagues conducted ethnobotanical research work in Toli Peer National Park, Azad Jammu and Kashmir, where they proved that EB uses increases with increasing number of plants and their results coincided with our findings [28,29]. Similar statistical tools were also applied in an ethnobotanical expedition conducted by Mehwish *et al*., 2019 on District Bhimber of Azad Jammu and Kashmir, Pakistan [30]. Similar results have been proved in past research works [52–54] which proves that rural area people still rely on wild flora for fulfilling the needs of their daily life and particularly female retain and use TIK more prevalently then male which is due to restricted life in rural and remote areas which may be because of cultural barriers or lack of resources in the areas.

**Table 7:** Spearman correlation for Male informants from Dawarian and Rati Gali, AJK, Pakistan.

Age	Number of species	*d* 1	Number of uses	*d* 2	*d = d* 2−*d* 1	*d*^2^
25	14	8	16	5	−3	9
35	9	2	4	1	−1	1
44	16	6	28	7	1	1
55	12	4	11	3	−1	1
66	7	1	10	2	1	1
85	18	7	20	6	−1	1
94	10	3	13	4	1	1

Sum of value of *d*^2^ = 15 $r_{\text{c}}\;=\;1-\frac{\left[6^{\sum {\text{d}}^{2}}\right]}{\text{n}\left({\text{n}}^{\text{2}}-1\right)};\;r_{\text{c}}\;=\;1-\frac{\left[6\times 15\right]}{7\left(7^{2}-1\right)};\;r_{\text{c}}\;=\;1-\frac{\left[90\right]}{7\left(49-1\right)};\;r_{\text{c}}\;=\;1-\frac{\left[90\right]}{7\left(48\right)};\;r_{\text{c}}\;=\;1-\frac{\left[90\right]}{336}$; *r*_c_ = 1−[0.267]; *r*_c_ = 1−0.267; *r*_c_ = 0.733.

**Table 8:** Spearman correlation for female informants from Dawarian and Rati Gali, AJK, Pakistan.

Age	Number of species	d 1	Number of uses	d 2	*d = d* 2−*d* 1	*d*^2^
24	11	2	13	1	−1	1
35	14	5	18	4	−1	1
45	18	7	20	6	−1	1
54	10	1	15	2	1	1
65	12	3	16	3	0	0
75	13	4	19	5	1	1
84	15	6	22	7	1	1

Sum of value of *d*^2^ = 6 $r_{\text{c}}\;=\;1-\frac{\left[6^{\sum {\text{d}}^{2}}\right]}{\text{n}\left({\text{n}}^{\text{2}}-1\right)};\;r_{\text{c}}\;=\;1-\frac{\left[6\times 6\right]}{7\left(7^{2}-1\right)};\;r_{\text{c}}\;=\;1-\frac{\left[36\right]}{7\left(49-1\right)};\;r_{\text{c}}\;=\;1-\frac{\left[36\right]}{7\left(48\right)};\;r_{\text{c}}\;=\;1-\frac{\left[36\right]}{336}$; *r*_c_ = 1−[0.107]; *r*_c_ = 1−0.107; *r*_c_ = 0.893.

Informant consensus factor (ICF) was used to support the data and to see the degree of agreement on each plant reported by informants (Table 9). The highest value (0.94) of ICF was for diseases group “tuberculosis and leucorrhea”, followed by stomachache and flatulence (0.93), diabetics and blood pressure (0.92) and asthma and chest infections (0.88) as shown in Table 9. The high values of ICF for Tuberculosis (TB), asthma and chest infections may be use of cold and high mountaineous house where smoke of burning of wood (used for fuel purpose to cook and heating purpose) causes lungs infirmities. Feminist disease leucorrhea’s high rate might be due to excessive eating of high energy (hot) foods to combat cold environment. The common occurrence of diabetics and blood pressure may be due to changes in life style and excessive uses of fat/ghee by the indigenous people. These findings are corroborate with previous research works [26,27]. The comprehensive ICF analysis depicted that similar types of infirmities were reported in other areas of AJK [53,56,65,66] and Pakistan [54,55,58,73–76].

**Table 9:** Informant consensus factor (ICF) for different diseases categories from Dawarian and Rati Gali, AJK, Pakistan.

Diseases	Species (nt)	All spp. %	Used citation (nur)	All citation %	$\text{ICF}\;=\;\frac{\left(\text{nur}-\text{nt}\right)}{\left(\text{nur}-1\right)}$
Cough and cold	16	12.03	125	11.92	0.88
Stomachache and flatulence	21	15.79	345	32.89	0.94
Asthma and chest infections	15	11.28	143	13.63	0.90
Joint and muscle pain	9	6.77	65	6.20	0.88
Fever and malaria	9	6.77	36	3.43	0.77
Epilepsy and mental disorders	9	6.77	33	3.15	0.75
Dysentery and bowls	19	14.29	53	5.05	0.65
Cardiovascular disorders	7	5.26	45	4.29	0.86
Snake and other bites	7	5.26	25	2.38	0.75
Kidney and urinary disorders	8	6.02	18	1.72	0.59
Diabetics and blood pressure	8	6.02	93	8.87	0.92
Tuberculosis and leucorrhea	5	3.76	68	6.48	0.94

The other common use of plants was fuel with ICF (0.83) purpose which is pivotal source for cooking and heating the rooms in chilling cold weather. The second was and thatching (ICF = 0.82) where people use plants or their parts for construction/thatching houses because people in study areas only depends on tree for houses/shelter formation. The lowest value is for fodder 0.18 (Table 10). Similar findings were correlated and strongly supported by Farooq and his colleagues [26]. Our both ICF results for ethnomedicines and ethnobotanical were coincidence with past researchers published by different scientists in rest of the world [30].

**Table 10:** Informant consensus factor (ICF) for different categories from Dawarian and Rati Gali, AJK Pakistan (for other purposes).

Category	Species (nt)	All spp. %	Use citation (nur)	All citation %	$\text{ICF}\;=\;\frac{\left(\text{nur}-\text{nt}\right)}{\left(\text{nur}-1\right)}$
Fodder	28	35.44	34	16.59	0.18
Food	14	17.72	17	8.29	0.19
Fuel	19	24.05	105	51.22	0.83
Furniture	9	11.39	14	6.83	0.38
Construction	5	6.33	17	8.29	0.75
House Thatching	4	5.06	18	8.78	0.82

According to direct matrix ranking (DMR) analysis was calculated to determine biotic pressure and conservation status of different plant species being used by indigenous people of the area. The data proved that *P*. *wallichiana* was most prevalently used (DMR = rank-1^st^) and it was under severe threats due to anthropogenic activities. *C*. *deodara* ranked 2^nd^ which is also used for fuel, construction and preferably for commercial purpose that may be smuggling of its valuable timber in local and national markets (Table 11). The third species was *P*. *roxburghii* which depicted that this plant is multifariously used for domestic and commercial needs and its wood being of high worth is also smuggled which created need of conservation. These findings were strongly justified by different taxonomists in various studies. They calculated DMR from various regions of the world as strongly correlated with our studies [35–40].

**Table 11:** Direct matrix ranking (DMR) of tree species with different uses other than medicinal value from Dawarian and Rati Gali, AJK, Pakistan.

Uses	*P*. *wallichiana*	*P*. *roxburghii*	*P*. *smithiana*	*C*. *deodara*	*A*. *pindrow*	*A*. *cappadocicum*	*P*. *alba*	*S*. *tetrasperma*
Construction	40	40	35	36	30	0	0	0
Hedging and Fencing	20	18	15	10	15	14	20	22
Fire wood	25	29	35	38	30	32	28	19
Cash income	40	38	30	35	20	0	2	0
Fodder	5	2	8	4	10	20	22	29
Fruit, Food	0	0	0	5	0	0	0	0
Total	130	127	123	128	105	66	72	70
Rankings	1^st^	3^rd^	4^th^	2^nd^	5^th^	8^th^	6^th^	7^th^

Thus, the current study is very useful and of high significance because it provides baseline primary data on WIPs being commonly used in various traditional ethnomedicines (TEMs). This research provides pivotal information for conservation of cultural diversity of comparatively isolated and remote areas of Neelam valley. This study also documents the phytodiversity of indigenous wild flora and domestic as well as commercial worth is mentioned. The research indicated that there is dare need toc conserve TEMs knowledge of area before it is diminished or eroded from the region. The study will also assist to initiate protection measures and conserve the near-to-threatened species as indicated in DMR analysis.

Through this study important and unique medicinal plants can be selected for further phytochemical studies to confirm their ethnopharmacological analysis and drug discovery. In study area, out of total 103 plants about 58 (56.31%) are the plants which have not been reported for any traditional ethnomedicine uses from Pakistan which proves the novelty of the research work. Albeit 27 plant species (26.21%) having reported in past studies for TEMs but in this research work very different traditional ethnomedicinal use-reports are documented (Table 12). It proves that area has unique biocultural diversity (BCD) and phytogeography as well as phytodiversity. These explorations are of high worth because reported first time in this study and it will provide valuable future research for drug discovery and development. The local people of the area primarily are dependent on wild resources for life necessities and it is coincided with past works cited in the literature, where it is proved that rural people majorly use wild plants for coping daily life needs [55–68].

**Table 12:** Novelty aspect analysis by comparing of ethnobotanical and ethnomedicinal uses of indigenous plants from Dawarian and Rati Gali, AJK (Pakistan).

S. No.	Species name	Already reported traditional ethnomedicinal uses	Newly reported ethnomedicinal uses
1	*Acer cappadocicum* Gled.	It is used as a fuel (Sher et al., 2011).	It is used as ethnomedicine to cure diabetes, dysentery and diarrhea.
2	*Ajuga bracteosa* Wall.	It is used for blood purification as cited by (Hussain et al., 2006). Used to treat abdominal pain as cited by (Ahmad et al., 2011).	The flower powder is used for cure of diabetes. The root tea is used for killing of stomach worms. Paste of leaf helpful to cure headache.
3	*Ajuga parviflora* Benth.	Nil	The plant leaf extract is used for cure of typhoid and malaria. The root decoction is used for cure of chronic fever and chest pains
4	*Allium griffithianum* Boiss.	It is used to cure cough as cited by (Khan et al., 2015).	It is used to cure fever. It is used as tonic for early digestion of food.
5	*Aconogonon alpinum* (All.) Schur MUH-1779	Leaves are used as food as cited by (Mahmood et al., 2011).	Root is used for the treatment of joints pain and tonic as wormicidal.
6	*Actaea spicata* L. MUH-1780	Nil	The leaf extract is used for curing of nerve infirmities, joints inflammation, leucorrhea and rheumatism.
7	*Aesculus indica* (Wall. ex Cambess.) Hook. MUH-1781	It is used as fuel as cited by (Sher et al., 2011).	The root powder is used for treatment of rheumatic pains. The bark extract is used for curing of headache.
8	*Aconitum heterophyllum* Wall. ex Royle MUH-1782	Roots are used to treat fever and vomiting as cited by (Hazrat et al., 2011). Used to treat fever as cited by (Kumar et al., 2009).	The root decoction is used as expectorant and febrifuge agent. The bark powder is used for cure of inflammation and chronic joints pains.
9	*Abies pindrow* Royle. MUH-1783	Nil	The paste of the leaf is applied on cuts wounds bruises to get rid of bacteria and germs. The root tea is used for cure of asthma and cough. Seeds decoction is used for treating fever, hyperglycemia and bronchitis.
10	*Achillea millefolium* L. MUH-1784	Nil	Paste prepared from this plant is used in stanching the flow of blood from wounds. Leaves are chewed to treat teeth pain. Leaf juice is poured in ear to treat ear pain. Plant is also used to treat T.B., stomach disorder and fever in form of Tea.
11	*Artemisia japonica* Thunb. MUH-1785	Nil.	The juice of leaves is used for cough and asthma.
12	*Anaphalis triplinervis* Clarke MUH-1786	Nil	The leaf decoction is used in cure of epilepsy. The whole plant paste is used for treating of animal feet diseases as ethnoveterinary medicines.
13	*Artemisia macrophylla* Fisch. ex Besser MUH-1787	Nil	The root powder is used for cure of brunt wounds. The flower is used to make admixture of flower with sugar and is used for cure of body tonic
14	*Astragalus graveolens* Benth. MUH-1788	Nil.	Leaf is used for cure of wounds. Fruit is eatable and used as antioxidant agent.
15	*Ajuga parviflora* Benth MUH-1789	Nil.	It is used as fodder.
16	*Adiantum aethiopicum* L. MUH-1790	Nil	Juice of leaves is used for the treatment of chest burning, stomachache and blood purification.
17	*Arisaema tortuosum* (Wall.) Schott MUH-1791	Tubers are appied over wound of snake bite as cited by (Swarnkar and Katewa, 2008).	The roots are used as wormicide. The extract of leaf is used to cure cattle worms and stomach issues.
18	*Astragalus chlorostachys* Bunge MUH-1792	Nil	The plant is used as fodder for the livestock and cattle.
19	*Bergenia ciliata* (Haw.) Sternb. MUH-1793	Nil	Extracts of leaves is used as earaches relieve while roots are used as a tonic in treatment of fevers, diarrhoea and pulmonary affections.
20	*Berberis lycium* Royle MUH-1795	Decoction of roots is used to treat internal wounds especially bone fractures as cited by (Mahmood et al., 2011).	Dried leaves are used for the treatment of headache, stomachache, joints pain and toothache.
21	*Bistorta amplexicaulis* (D.Don) Greene MUH-1796	Plant is used for making tea as cited by (Qureshi et al., 2007).	Dried root is used as tea to cure stomachache. The herbaceous roots are tonic for enhancing of cow milk. The root decoction is used for cure of toothache.
22	*Buddleja crispa* Benth. MUH-1797	Plant is used as fuel as cited by (Irfan et al., 2018).	The root infusion is used for curing wound healing by increasing platelets. Its leaf extract is used for inflammation and analgesic purpose.
23	*Buxus wallichiana* Baill. MUH-1798	Nil	Dried leaves are used in the treatment of joints pain and muscles pain.
24	*Convolvulus arvensis* L. MUH-1799	It is used as fodder as cited by (Zabiullah et al., 2006).	Leaf is used as vegetable which is purgative and laxative. The stem paste is used for treating of joints pain
25	*Cirsium arvense* (L.) Scop. MUH-1800	Nil	Powdered form mix with water is used as tonic.
26	*Campanula pallida* Wall. MUH-1801	Nil	The root decoction is used for treating scabies.
27	*Cynoglossum lanceolatum* Forssk. MUH-1802	Plant powder is used as laxative as cited by (Amjad et al., 2015).	The foliar past is applied on abscess to remove pus. It is also use in asthma.
28	*Cuscuta reflexa* Roxb. MUH-1803	Nil	Juice of the whole plant used to increase the length of hairs and make strong. Its decoction is used in jaundice and cure of spleen disorders. The infusion is used for treating urinary issues.
29	*Cedrus deodara* (Roxb. ex D.Don) G.Don MUH-1804	Oil of wood is used for skin diseases as cited by (Ishtiaq et al., 2013).	Oil of wood is used for toothache. Wood is also used as fuel. The leaf decoction is used for treating of piles. The root burnt used to cure epilepsy.
30	*Corylus colurna* L. MUH-1806	Nil	The leaf extract is used as antioxidant. Leaf extract is useful as cure of snake poison.
31	*Corydalis vaginans* Royle MUH-1807	Nil	The sap of the plant is used in the treatment of eye diseases.
32	*Cotoneaster microphyllus* Wall. ex Lindl. MUH-1808	Nil	The leaf decoction is used for treating of diarrhoea. The root powder is used as effective to cure wounds.
33	*Corydalis govaniana* Wall. MUH-1809	Nil	Juice of leaves is used for the treatment of fever and skin problem.
34	*Caltha alba* Cambess. MUH-1810	Nil	Dried powdered or juice of this plant is used to reduce muscle pain and sedative.
35	*Cenchrus pennisetiformis* Steud. MUH-1811	Used as fodder for cattle as cited by (Chaudhari et al., 2013).	The leaf extract is used for cure of bacterial infections. It is used as fodder for cattle and rodents.
36	*Clinopodium vulgare* L. MUH-1812	Nil	A sweet and aromatic herb tea is made from the fresh leaf for cure of headache and migraine pain.
37	*Erysimum hieraciifolium* L. f. MUH-1814	Nil	The leaf decoction is used for cure of foot rot. The root infusion is used for treatment of pimples and bruises on legs.
38	*Erysimum hedgeanum* Al-Shehbaz MUH-1815	Nil	The juice of whole plant is use to kill lices in animals.
39	*Euonymus hemsleyanus* Loes. MUH-1816	Nil	The leaf decoction is used as tonic for hair growth. It is used as fodder cattle and rodents.
40	*Elsholtzia strobilifera* (Benth.) Benth. MUH-1817	Nil	The root infusion is used for treating indigestion, flatulence and diarrhea. The stem bark is used for cure of pharyngitis disorders.
41	*Fragaria nubicola* Lacaita MUH-1818	Fruit is edible as cited by (Qureshi et al., 2007).	The leaf decoction is used for curing of blemishes infirmities. The fruit extract with milk is used for damaged and broken nerve disorders..
42	*Geranium rotundifolium* L. MUH-1819	The dried roots were grinded, sugar and milk are added in it, and then used for pain relief of joints as cited by (Ahmed et al., 2013).	The dried roots were grinded, sugar and milk are added in it, and then used for pain relief of joints. The root decoction is used to cure epilepsy
43	*Geranium villosum* Ten. MUH-1820	Nil	It is used as food for cure of edema.
44	*Gerbera gossypina* (Royle) Beauverd MUH-1821	Nil	Root paste is applied to wounds to control bleeding.
45	*Hylotelephium ewersii* (Ledeb.) H.Ohba MUH-1822	Nil	It is believed to be having cooling effect if the juice of the leaves mix with water and drink.
46	*Indigofera heterantha* Brandis MUH-1824	Shoots are used as fodder, branches as ropes, brooms and fuel as cited by (Hazrat et al., 2011).	The leaf decoction is used for cure of stomach disorder and abdominal pains.
47	*Isodon rugosus* (Wall.) Codd MUH-1825	Nil	Juice of the leaves is used for stomachache.
48	*Juniperus communis* Brand. MUH-1827	Nil	The decoction of root is used for cure of inflammation and diarrhea. The leaf extract is used as microbicide and antiseptic.
49	*Lespedeza juncea* (L.f.) Pers. MUH-1828	Nil	The decoction of root is used as cure of diarrhea and dysentery. The leaf tea is used for stomach pains.
50	*Ligularia thomsonii* Clarke. MUH-1829	Nil	Dried root or powdered of root is used in the treatment of asthma, stimulate blood flow, reduce inflammation and stopping cough.
51	*Mentha longifolia* L. MUH-1830	Used to cure stomach disorders as cited by (Kilic et al., 2013).	Shoot is used for gas trouble. Juice of leaves expels worms from the stomach. It is also as condiment.
52	*Matricaria chamomilla* L. MUH-1831	Nil	Root powder is used for toothache. The leaf decoction is used in relief of fever and inflammation.
53	*Meliosma simplicifolia* (Roxb.) Walp. MUH-1833	Nil	Leaf decoction is used as cure of inflammation reducer of legs and broken joints.
54	*Oxalis corniculata* L. MUH-1834	Nil	Juice of leaves and flowers mixed together is used for the treatment of eyes.
55	*Onychium japonicum* (Thunb.) Kunze MUH-1835	Nil	It is used as vegetable. Dried root or powdered root is used for the treatment of asthma and flu.
56	*Onosma bracteata* Wall. MUH-1837	Leaf infusion is taken for stomachache as cited by (Rashid et al., 2018).	Powder of dry root is used against asthma and bronchitis. Decoction of leaf is given in stomach and bladder irritation.
57	*Origanum vulgare* L. MUH-1838	Nil	It is used for muscles pain, cold and toothache. It is also as vegetable and fodder.
58	*Polygala chinensis* L. MUH-1839	Nil	This plant is used for treatment of snake bites.
59	*Pedicularis brevifolia* D.Don MUH-1841	Nil	Powdered leaf is used for the treatment of cough, fever, asthma and skin disease. Dried or powdered root is used for the treatment of stomachache.
60	*Primula denticulata* Sm. MUH-1842	Nil	Juice of stem is used for eye diseases.
61	*Podophyllum hexandrum* Royle MUH-1843	Nil	Powdered leaf is used in the treatment of asthma. It is also used to reduce bulb in throat.
62	*Populus alba* L. MUH-1844	Used as a fuel as cited by (Khan and Khatoon, 2007).	The leaf decoction is used to cure gout, joint pain and arthritis. The root infusion is used for backbone and lumber pains.
63	*Plantago lanceolata* L. MUH-1845	Nil	The root tea is used for cure of cold, flu and fever. The bark extract is employed is used for cure of debility and body general weakness.
64	*Persicaria mitis* (Schrank) Holub MUH-1846	Nil	Tea is made by root which help to reduce the joints pain.
65	*Podophyllum emodi* Wall. ex Hook.f. & Thomson MUH-1848	Nil	The root tea is used to cure colds, fever and cough. The bark powder is used for cure of wounds.
66	*Pinus wallichiana* A.B.Jacks. MUH-1849	Wood is used for construction purposes, seeds are edible and cones are used as fuel as cited by (Sinha, 2019).	Smell of resin reduce severe cough. Powder of leaf and bark used with cold water useful for dysentery.
67	*Pinus roxburghii* Sarg. MUH-1850	Wood is used for furniture and fuel as cited by (Zabiuhullah, 2006).	Powder of leaf and bark is used with cold water for dysentery. Smoke is used to repel the mosquitoes and other insects.
68	*Rosa macrophylla* Lindl. MUH-1851	Nil	Fruit is used in fever to cure from it.
69	*Rheum emodi* Wall. MUH-1852	Leaves are used as vegetable as cited by (Khan et al., 2015).	The powdered root and stem mix together with hot water to relieve constipation.
70	*Rubus niveus* subsp. *horsfieldii* (Miq.) Focke MUH-1853	Nil	The leaf decoction is used for cure of debility and menstrual disorders. The root extract is used to treat eye problems.
71	*Rheum australe* D. Don MUH-1854	Leaves are used as vegetable and root is used to treat wounds as cited by (Mahmood et al., 2011).	Paste of root is used for wound healing.
72	*Rhus succedanea* L. MUH-1855	Used as fuel as cited by (Mahmood et al., 2011).	The root extract is used as antidote for scorpion sting. The root infusion is applied for as febrifuge and antivinous.
73	*Sorghum halepense* Pers. MUH-1859	Used as fodder as cited by (Ahmad et al., 2011).	Juice of root is used for the asthma.
74	*Senecio chrysanthemoides* DC. MUH-1860	Nil	Leaf decoction is used for cure of rashes and bruises. Root paste us used for scorpion sting antidote.
75	*Skimmia laureola* Franch. MUH-1861	Nil	Tea is made by dry leaves which is very effective in joints pain, muscles pain, stomach pain and bone pain. Powdered leaves also used in deserts.
76	*Symplocos paniculata* (Thunb.) Miq. MUH-1863	Nil	Powdered leaf is used in the treatment of menorrhagia, eye disease.
77	*Sarcococca saligna* Müll.Arg. MUH-1864	Nil	Powdered leaf is used in constipation, blood purification and muscles relaxation.
78	*Satyrium nepalense* D.Don MUH-1865	Used as tonic and to cure dysentery and malaria as cited by (Pant and Samant, 2010).	Tubers are used as tonic and to cure dysentery and malaria fever.
79	*Scutellaria linearis* Benth. MUH-1866	Nil	Powdered leaf is used to reduce inflammation and diarrhea.
80	*Swertia paniculata* Wall. MUH-1867	Nil	Leaf extract is used to cure hepatic disorders. The root decoction is used to treat diabetes.
81	*Solidago capitata* Fisch. ex Herder MUH-1868	Nil	Powdered plant is used to heal wounds.
82	*Thymus linearis* Benth. MUH-1869	Nil	Tea is made by this plant which help to reduce fats in body, abdominal pain and gas trouble.
83	*Taxus baccata* L. MUH-1870	Nil	The leaf extract is used to treat cold and fever. The root powder is used for treatment of cough and chest pains. It is also used for preparation of taxol medicines.
84	*Viola biflora* L. MUH-1872	Nil	Leaves are used as vegetables. Tea is made by dry leaf which helps in cough headache and flu.
85	*Viscum album* L. MUH-1875	Nil	Powdered leaves are used in the treatment of cough and asthma.
86	*Valeriana jatamansi* Jones MUH-1876	Nil	Powdered root is used for the treatment of joints pain. It is also used in sweet dishes.
87	*Viola canescens* Wall. MUH-1877	Flowers and leaves are used to treat cough as cited by (Gilani at al., 2006).	Powder of leaf and flowers is given internally in the treatment of coughs and asthma.
88	*Wulfenia amherstiana* Benth. MUH-1878	Nil.	Root decoction us used to cure kidney disorders.

The results indicated that many species are first time reported from the study area and these are novel reporting and documentation of ethnomedicinal uses. The collected data will be helpful in future drug discovery and drug development. Many Similar type of justifications for conducting such type of ethnobotanical research proves clues and directives for further research to discover neo-drugs and development and in this research there is also huge scope for drug discovery [66–72]. The plants are play pivotal role in daily of human being because they provide all fundamental needs of man, animals, birds and other microbes as well. The ecosystem services can only proceed if the plants are present in good number (population) otherwise there will be shrinkage and stoppages of ecosystem workings in any part of the earth or biosphere. This will also change the life of indigenous people of any area in the world. The plants provide mainstream pathway for their use to cure infirmities of man and livestock as well. The plants are producers with role in life sustenance for the human being in form of food, forage, fodder, fuel, timber and medicines provisions to meet the life necessities of indigenous communities [73–76]. Hence, this study will be very fruitful to document the ethnobotanical uses and explore their potential for drug production and also devise the conservation status of various plants for future use. It will also assist to preserve TEK of folklore cultural diversity and conserve near to threatened species.

### Conclusion

The present research was focused to explore the various ethnobotanical uses of plants from unexplored areas Dawarian and Rati Gali of District Neelam, Azad Jammu and Kashmir using quantitative ethnobotanical tools. This research was carried out by interviewing the local peoples through a questionnaire method using structured and semi-structured procedure. The analytical tools proved which plants have more medicinal potential than other and recommend the further ethnopharmacological analysis to discover drug. Local peoples use indigenous wild plants to cure different diseases like asthma, dysentery, cancer, diabetes, epilepsy, cardiovascular disorders, constipation, cold, fever, stomachache, joint pain, arthritis, wound healing, kidney infection and skin diseases. About 58 (56.31%) plants species are hitherto not reported for their TEMs use from Pakistan and elsewhere and hence, reported first time which make this study valuable for further ethnopharmacological research to discover new drugs. Whereas 27 (26.21%) plants TEMs are described here which are prior not published and these novel in the research. So, this study will be useful those for the local peoples and researchers in different fields such as ethnopharmacology, agriculture, phytochemistry, pharmacy, biotechnology and conservationists for future work. Moreover, this study recommends the future phytochemical analysis to authenticate the bioconstituent which may be used for novel drug formation to cope the MDR bacteria and other microbial infirmities.
